The article "N6-Methyladenosine Reader YTHDF2 Enhances Non-Small-Cell Lung Cancer Cell Proliferation and Metastasis through Mediating circ_SFMBT2 Degradation" was published in 2022. Journal: Contrast Media Mol Imaging.

# N6-Methyladenosine Reader YTHDF2 Enhances Non-Small-Cell Lung Cancer Cell Proliferation and Metastasis through Mediating circ_SFMBT2 Degradation

**DOI:** 10.1155/2022/1087622

**Published:** 2022-07-16

**Authors:** Jing Xu, Yan Shang, Xiong Qin, Yun Gai, Feng Cai, Hua Xiao, Chen Zhou, Youhui Fu, Xiahui Ge

**Affiliations:** ^1^Department of Respiratory Medicine, Seventh People's Hospital of Shanghai University of TCM, Shanghai 200137, China; ^2^Department of General Practice, Changhai Hospital, Naval Medical University (Second Military Medical University), Shanghai 200433, China; ^3^Department of Respiratory and Critical Care Medicine, Changhai Hospital, Naval Medical University (Second Military Medical University), Shanghai 200433, China; ^4^Department of Thoracic Surgery, Shanghai Pulmonary Hospital, Tongji University School of Medicine, No. 507, Zhengming Road, Shanghai 200433, China; ^5^Department of Oncology, Seventh People's Hospital of Shanghai University of TCM, Shanghai 200137, China

## Abstract

**Objective:**

circ_SFMBT2 was reported to facilitate malignant progression in various cancers, but its function in non-small-cell lung cancer (NSCLC) has not been fully uncovered. This study aimed to investigate the effects of N6-methyladenosine (m6A) methylation of circ_SFMBT2 (circ_0017628) on non-small-cell lung cancer (NSCLC) and its underlying mechanisms.

**Methods:**

Paired tumor and noncancerous tissues from NSCLC patients were surgically collected from January 2020 to March 2021 in our hospital. The levels of circ_SFMBT2 and LATS2 in NSCLC and human bronchial epithelial cells were assayed with qRT-PCR. Overexpression or silencing of circ_SFMBT2, LATS2, or YTHDF2 was performed in the NSCLC cells. CCK-8, colony-forming, and transwell assays were performed to analyze cell proliferation, viability, and migration, respectively. Meanwhile, the expression of MMP-9, E-cadherin, vimentin, and the Hippo/YAP pathway components was examined by western blotting. The m6A enrichment in circ_SFMBT2 was verified using methylated RNA immunoprecipitation, and interaction between circ_SFMBT2 and YTHDF2 was assessed by RNA pull-down and immunoprecipitation assays.

**Results:**

Both circ_SFMBT2 and LATS2 were lowly expressed in NSCLC cells and tissues. A positive correlation of circ_SFMBT2 with LATS2 was identified, and circ_SFMBT2 was localized predominantly in the cytoplasm. circ_SFMBT2 overexpression negatively regulated cell proliferation, viability, migration, and epithelial-mesenchymal transition while promoting the Hippo/YAP pathway activation. Notably, knockdown of LATS2 effectively abrogated the inhibitory effects of circ_SFMBT2 overexpression on NSCLC cell malignancies. Besides, m6A was specifically enriched in circ_SFMBT2, and circ_SFMBT2 could bind to YTHDF2. Silencing of YTHDF2 led to an increase in circ_SFMBT2 expression while inhibiting the malignancy of cancer cells.

The article "N6-Methyladenosine Reader YTHDF2 Enhances Non-Small-Cell Lung Cancer Cell Proliferation and Metastasis through Mediating circ_SFMBT2 Degradation" was published in 2022. Journal: Contrast Media Mol Imaging.

**Conclusion:**

Our results showed that YTHDF2 could facilitate NSCLC cell proliferation and metastasis via the Hippo/YAP pathway activation by mediating circ_SFMBT2 degradation.

## 1. Introduction

Lung cancer is the most prevalent cause of cancer-associated deaths worldwide, with 1.6 million deaths yearly and 240,000 new cases in 2020 [1]. An estimated 85% of all lung cancer patients suffer from non-small-cell lung cancer (NSCLC) [2]. NSCLC treatment varies for each stage of the disease. Although significant advancements have been made in chemotherapy, radiotherapy, surgery, and targeted therapy, NSCLC patients have a 5-year survival rate as low as 16.6% [3]. Due to its multifocality and complexity, NSCLC is linked to a high risk of recurrence even following multimodal treatment [4]. Thus, pathogenetic studies of NSCLC may contribute to innovative and effective treatments of the patients, as well as the identification of new and important diagnostic markers.

Circular RNAs (circRNAs) are a group of noncoding RNAs harboring a covalently closed-loop conformation, which is generated from the reverse clipping of exonic mRNAs (pre-mRNAs) [5]. circRNAs are implicated in various pathophysiological processes, such as brain development and tumorigenesis [6]. Meanwhile, circRNAs have been found to function in numerous cancers, suggesting that they may potentially serve as a biomarker or therapeutic target. In these cases, an elevated level of circPRKCI, namely E2F7, ultimately promotes lung adenocarcinoma development by competing for binding to miR-545 and miR-589 [7]. circTP63 competes for binding to miR-873-3p and upregulates FOXM1 to expedite cell proliferation in lung squamous cell carcinoma [8]. circ_SFMBT2, a newly discovered circRNA with a circular structure, is derived from the SFMBT2 gene [9, 10]. It has been reported that circ_SFMBT2 positively regulates gastric cancer cell proliferation via the miR-182-5p/CREB1 axis [11]. circ_SFMBT2 has also been demonstrated to facilitate the malignant phenotype of esophageal cancer through regulating SLC1A5 in a miR-107-dependent manner [9]. To date, the function of circ_SFMBT2 in NSCLC cell development remains largely unknown.

As the most abundant modification in mRNAs, N6-methyladenosine (m6A) constitutes over 80% of all RNA modifications [12]. Strikingly, m6A is involved in the quantitative and qualitative regulation of target RNAs by modulating RNA splicing, stability, translocation, and translation [13]. Aberrant m6A methylation could cause dysregulation of genes that are essential for controlling key cellular processes while disrupting homeostasis, thus incurring disorders. Of note, m6A reader YTHDF2 mainly regulates splicing events and post-transcription in the cytoplasm. YTHDF2 can also transport mRNAs from actively translated mRNA repertoires to decaying mRNA repertoires, resulting in mRNA degradation [14]. Besides, studies have found that YTHDF2 facilitated malignant progression in several cancers, including early NSCLC; in this case, its elevated expression was linked with tumor growth and metastasis [15]. Other studies have suggested the potential of YTHDF1 and YTHDF2 as new prognostic factors and drug targets associated with the tumor immune microenvironment of NSCLC [16]. However, it should be noted that YTHDF2 was found to play opposite roles in different types of cancers as well. For instance, it was shown to be upregulated and acted as an oncogene in cancers including acute myelocytic leukemia (AML), lung cancer, and gastric cancer [PMID: 31711642, 31031138, and 31504235], while its overexpression in osteosarcoma and melanoma was associated with decreased cancer cell proliferation and migration (PMID: 31239444 and 32021563). Currently, the biological role of YTHDF2 in NSCLC has not yet been fully uncovered.

The article "N6-Methyladenosine Reader YTHDF2 Enhances Non-Small-Cell Lung Cancer Cell Proliferation and Metastasis through Mediating circ_SFMBT2 Degradation" was published in 2022. Journal: Contrast Media Mol Imaging.

In this study, we performed in vitro experiments to elucidate the relationship between YTHDF2 and circ_SFMBT2 and further characterized their roles in NSCLC to provide new information that could lead to the identification of new biological targets and development of strategies for improving the clinical treatment of NSCLC.

## 2. Materials and Methods

### 2.1. Tissue Specimens

Paired tumor and normal tissues from NSCLC patients were surgically collected from January 2020 to March 2021 at our hospital. All the patients voluntarily provided written informed consent. Ethical approval was granted by the ethics committee of our hospital (2020-IRBQYYS-011). All experiments described as follows were repeated three times.

### 2.2. Cell Culture and Transfection

NSCLC cells (A549, H460, H1299, and H1650) or human bronchial epithelial (HBE) cells were grown in DMEM medium (Gibco, USA) with 10% FBS, penicillin (100 mg/mL), and streptomycin (10 mg/mL) at 37°C under 5% CO_2_. A549 or H1299 cells were transfected with negative vector, circ_SFMBT2 overexpression vector (circ_SFMBT2), YTHDF2 siRNA (si-YTHDF2), LATS2 siRNA (si-LATS2), and negative plasmid (siNC), respectively, following the instructions of the Lipo 2000 reagent. After 6 h of transfection, the medium was substituted with a fresh medium, and the culture was continued for 48 h for subsequent experiments.

The article "N6-Methyladenosine Reader YTHDF2 Enhances Non-Small-Cell Lung Cancer Cell Proliferation and Metastasis through Mediating circ_SFMBT2 Degradation" was published in 2022. Journal: Contrast Media Mol Imaging.

### 2.3. Quantitative Reverse Transcription

PCR (qRT-PCR) Nuclear-cytoplasmic fractionation was performed using a nucleoplasmic isolation kit, and total RNA extraction from nuclei, cytoplasm, whole cells, or tissues was conducted using TRizol (Thermo, USA). Total RNA was subjected to detecting the concentration and purity by using NanoDrop and subsequently reverse transcription using a random primer reverse transcription kit. After that, cDNA was PCR-amplified with TaKaRa SYBR Green kit using the corresponding primers. A total of six replicates of the experiment was carried out. The expression of target genes was normalized to that of GAPDH, and the relative expression was determined using the 2−ΔΔCt method. The PCR primer sequences are presented in Table 1.

### 2.4. Fluorescence In Situ Hybridization (FISH)

FISH was carried out using the circ_SFMBT2-targeting probe. After 15 mins of fixation with 4% paraformaldehyde, the cells were washed with PBS and dehydrated in graded alcohols. Then, the cells were mixed with denatured DNA probes and hybridized overnight at 37°C in a humid and dark environment. On the following day, the cells were subjected to washing with saline-sodium citrate buffer thrice for 5 min each and blocked for 1 h in PBS with 1% BSA and 3% normal goat serum, followed by incubation with an antibiotin antibody (HRP-conjugated) overnight at 4°C. The images were acquired by using a fluorescent microscope.

### 2.5. Cell Counting Kit-8 (CCK-8) Assay

Cell proliferative ability was evaluated using the CCK-8 assay. The cells (5 × 10^3^/well) were seeded in a 96-well plate. After 24 h of culture, 10 *μ*L of the CCK-8 solution was applied to each well, and the plate was subjected to incubation at 37°C for 1 h. The OD values were determined at 450 nm.

### 2.6. Colony-Forming Assay

The cells were trypsin-digested, resuspended with a DMEM-complete medium, plated in a 6-well plate at a density of 7 × 10^2^ cells/well, and grown at 37°C with 5% CO2 for 14 days. When the colonies were visible, the cells were fixed in 4% paraformaldehyde, followed by staining using 0.1% crystal violet. The staining was photographed by using an inverted microscope, and the colonies with a single clonal cell number greater than 50 were counted. The colony formation rate was measured based on the following formula: (number of colonies/number of cells plated) × 100%.

### 2.7. Transwell Assays

Matrigel was thawed in a refrigerator for no less than 12 h, diluted in serum-free cell culture medium at 1 : 8, and spread in the transwell upper chamber at 4°C. The cells were harvested by trypsin digestion, resuspended with serum-free medium, and adjusted to a density of 1 × 10^5^ cells/ml. Subsequently, 100 *μ*L cells were applied into the upper chamber coated with or without Matrigel, respectively, while 700 *μ*L of 10% FBS-containing medium was added to the lower chamber. Transwell inserts were removed after 24 h of growth under 5% CO_2_ at 37°C, and the cells were then washed thrice with PBS. Thereafter, the cells were subjected to 30 min fixation, dried, and stained using 0.1% crystal violet for 30 min. Lastly, the stained cells were washed with PBS, dried, and examined using an upright microscope in randomly selected fields. Three visual fields were randomly selected for counting the positive cells.

The article "N6-Methyladenosine Reader YTHDF2 Enhances Non-Small-Cell Lung Cancer Cell Proliferation and Metastasis through Mediating circ_SFMBT2 Degradation" was published in 2022. Journal: Contrast Media Mol Imaging.

### 2.8. Western Blot Analysis

Tissues or cells were lysed in cell lysis buffer (Gibco, USA), and lysates were subjected to centrifugation (14,000 rpm for 15 min) at 4°C. Proteins were quantified using the BCA assay. Each protein sample (20 *μ*g) was separated on SDS-PAGE and electroblotted onto membranes. The membrane was blocked for 1 h in 5% nonfat dry milk and then incubated overnight at 4°C with specific primary antibodies. The following day, the membrane was washed and then subjected to 1 h of incubation with fluorescence-conjugated secondary antibodies at RT. The blot was developed with chemiluminescence reagents, and an imaging system was used to collect the images. Quantification of the immunoreactive bands was conducted using the Image J software, and the expression level of targets was normalized to that of GAPDH.

### 2.9. Methylated RNA Immunoprecipitation (MeRIP)

PBS-washed cells were collected, and total RNA was extracted with 2 ml QIAzol (QIAGEN, Germany). Then, 100 *μ*g of the total RNA was diluted in IPP buffer (150 mM NaCl, 10 mM Tris, pH 7.4, and 0.1% NP-40) with 10 *μ*g of the anti-m6A antibody to 300 mL. After 2 h of incubation at 4°C, the mixture was incubated with 50 *μ*L of Invitrogen G-conjugated Dynabeads for another 2 h. Thereafter, the beads were subjected to five washings using IPP buffer, followed by resuspension in 500 *μ*L QIAzol. Finally, the immunoprecipitated RNA fragments were purified and analyzed by qRT-PCR according to QIAzol's instructions. To observe m6A enrichment in circ_SFMBT2, both beads alone and isotype IgG-conjugated beads were included as a negative control.

### 2.10. RIP

Harvested cells were formaldehyde-treated, resuspended in nuclei isolation buffer, and lysed for 20 min at 4°C. After 15 min of centrifugation at 2500 g, the nuclear pellets were resuspended in RIP buffer, sonicated, and subjected to incubation with the anti-Ago2 or anti-IgG antibody overnight at 4°C in a shaker. The next day, proteinA/G beads were applied, and the incubation was continued for 1 h. Then, the beads were pelleted, washed, and subjected to RNA purification. The immunoprecipitated RNA samples were subjected to qRT-PCR assay to determine how circ_SFMBT2 could bind to YTHDF2.

The article "N6-Methyladenosine Reader YTHDF2 Enhances Non-Small-Cell Lung Cancer Cell Proliferation and Metastasis through Mediating circ_SFMBT2 Degradation" was published in 2022. Journal: Contrast Media Mol Imaging.

### 2.11. RNA Pull-Down Experiment

The biotinylated circ_SFMBT2 probe was obtained from GenePharma (Shanghai, China). C-1 beads (Life Technologies, USA) were coated with the circ_SFMBT2 probe by incubation with the probe for 2 h at RT. In the meantime, the harvested cells were lysed and incubated overnight at 4°C with the circ_SFMBT2 probe or oligo probe. The RNA complexes were isolated using an RNeasy mini kit. YTHDF2-induced enrichment of circ_SFMBT2 was assessed using qRT-PCR.

### 2.12. RNase R Digestion

Total RNA was isolated from the transfected cells. Then, 3 *μ*g of the extracted RNA was subjected to 30 min incubation with 20 U/*μ*L RNase R at 37°C. Afterward, qRT-PCR was conducted to quantify both circ_ and linear SFMBT2.

### 2.13. Determination of Actinomycin D

The cells were treated with actinomycin D for 0, 4, 8, 12, and 24 h, respectively. After incubation, the cells were harvested and subjected to total RNA extraction. circ_SFMBT2 expression in the cells was quantified using qRT-PCR.

### 2.14. Statistics

Statistical analysis was performed using the SPSS 26.0 software. All data were presented as mean ± SD. Comparison between multiple groups or two groups was made using one-way analysis of variance or the independent-sample *t*-test. The expression correlation between circ_SFMBT2 and LATS2 was assessed by Pearson's correlation analysis. *P* < 0.05 was indicative of statistical significance.

## 3. Results

### 3.1. circ_SFMBT2 Was Significantly Downregulated in NSCLC Cells and Tissues

We first analyzed circ_SFMBT2 expression in NSCLC tissue specimens using qRT-PCR. As depicted in Figure 1(a), circ_SFMBT2 expression was markedly reduced in the tumor tissues compared to their nontumor counterparts. Likewise, circ_SFMBT2 expression was decreased in the NSCLC cells, with A549 and H1299 cell lines exhibiting the lowest expression level (Figure 1(b)). Meanwhile, we observed that circ_SFMBT2 expression was significantly increased in the cytosol relative to the nucleus (Figures 1(c) and 1(d)). Moreover, the FISH assay revealed a predominant cytoplasmic localization of circ_SFMBT2 (Figure 1(e)). These results were indicative of an involvement of circ_SFMBT2 in NSCLC.

### 3.2. circ_SFMBT2 Inhibited Malignant Progression of NSCLC Cells by Upregulating LATS2 Expression

Given the vital function of LATS2 in NSCLC, this study further examined the possible effects of LATS2 on circ_SFMBT2 in NSCLC progression. As illustrated in Figures 2(a) and 2(b), the expression of LATS2 was markedly reduced in NSCLC cells and tissues compared to the controls, with the lowest level being in A549 and H1299 cells. Clearly, we observed a high expression of circ_SFMBT2 in the transfected cells, indicative of a successful transfection of the NSCLC cells with circ_SFMBT2 (Figure 2(c)). Of note, LATS2 was upregulated in the cells overexpressing circ_SFMBT2 (Figure 2(d)). Further analysis identified a positive correlation between circ_SFMBT2 and LATS2 (Figure 2(e)). To investigate the functional relationship between circ_SFMBT2 and LATS2, LATS2 was silenced in the cells overexpressing circ_SFMBT2, and malignant cell behaviors were analyzed. Strikingly, overexpression of circ_SFMBT2 significantly decreased the cell proliferative rate, viability, and migratory capability, while LATS2 knockdown in the circ_SFMBT2-overexpressing cells restored the *in vitro* malignant behaviors of NSCLC cells (Figures 2(f)–2(i)). Moreover, expression analysis of epithelial-mesenchymal transition-associated markers showed that circ_SFMBT2 overexpression led to an upregulation of MMP-9 and vimentin while downregulating E-cadherin. Notably, coexpression of circ_SFMBT2 and si-LATS2 restored the expression level of MMP-9, vimentin, and E-cadherin in the NSCLC cells (Figure 2(j)). These observations suggested that circ_SFMBT2 negatively could regulate NSCLC cell malignancy by upregulating LATS2.

The article "N6-Methyladenosine Reader YTHDF2 Enhances Non-Small-Cell Lung Cancer Cell Proliferation and Metastasis through Mediating circ_SFMBT2 Degradation" was published in 2022. Journal: Contrast Media Mol Imaging.

### 3.3. circ_SFMBT2 Participated in Regulating Hippo/YAP Pathway Activation in NSCLC Cell Lines

To investigate how circ_SFMBT2 affects the malignant behavior of NSCLC cells, we examined the Hippo/YAP pathway component expression in the cells. Western blotting revealed marked upregulation of LATS2 and LATS1 as well as a significant downregulation of YAP in the circ_SFMBT2 group compared with the vector group. Strikingly, the altered expression of LATS1 and YAP in circ_SFMBT2-overexpressing NSCLC cells was reversed by si-LATS2 treatment (Figure 3). Taken together, these data suggested that circ_SFMBT2 could affect NSCLC cell malignancy by activating the Hippo/YAP pathway.

### 3.4. YTHDF2 May Accelerate the Degradation of m6A-Modified circ_SFMBT2

To further investigate the mechanism underlying the low expression of circ_SFMBT2 in NSCLC cells, we predicted the m6A locus in circ_SFMBT2 by using the sequence-based SRAMP database of m6A modification site predictors (https://www.cuilab.cn/sramp). Notably, circ_SFMBT2 could be retrieved at multiple methylation sites of m6A (Figure 4(a)). As shown in the MeRIP assay (Figure 4(b)), circ_SFMBT2 was specifically enriched by the anti- m6A antibody. Moreover, circ_SFMBT2 was markedly upregulated in NSCLC cells with a reduced expression of the m6A reader YTHDF2 (Figures 4(c) and 4(d)). Meanwhile, RNA pull-down experiments revealed that YTHDF2 could recognize and bind to circ_SFMBT2 (Figure 4(e)). Besides, the RNA stability assay showed that the circ_SFMBT2 level in the YTHDF2 knockdown cells significantly declined over time, while the level at each time point was markedly elevated in the si-YTHDF2 group compared with the siNC group (Figure 4(f)). The abovementioned findings indicated that YTHDF2 could positively regulate the degradation of m6A-modified circ_SFMBT2.

The article "N6-Methyladenosine Reader YTHDF2 Enhances Non-Small-Cell Lung Cancer Cell Proliferation and Metastasis through Mediating circ_SFMBT2 Degradation" was published in 2022. Journal: Contrast Media Mol Imaging.

### 3.5. Silencing circ_SFMBT2 Reversed Tumor Suppression in YTHDF2-Knockdown NSCLC Cells

To clarify the relationship between circ_SFMBT2 and YTHDF2 and their roles in NSCLC progression, we performed functional assays in cells with a reduced expression of YTHDF2 or both circ_SFMBT2 and YTHDF2. As shown in Figures 5(a)–5(d), knockdown of YTHDF2 remarkably decreased the cell proliferative rate, viability, and migration ability, while cosilencing of circ_SFMBT2 and YTHDF2 restored the malignant behaviors of the NSCLC cells. Moreover, western blotting revealed a decreased expression of MMP-9, vimentin, and YAP, along with an upregulation of E-cadherin, LATS2, and LATS1 in the YTHDF2-knockdown cells. Notably, silencing circ_SFMBT2 in the YTHDF2-knockdown cells significantly reversed the expression levels of MMP-9, vimentin, YAP, E-cadherin, LATS2, and LATS1 (Figures 5(e) and 5(f)). These observations suggested that circ_SFMBT2 knockdown significantly attenuated the inhibitory effect of si-YTHDF2 on NSCLC progression.

## 4. Discussion

An increasing body of evidence shows that circRNA expression correlates with clinicopathological features of cancer patients [17]. The present study found that both circ_SFMBT2 and LATS2 were markedly downregulated in NSCLC cells and tissues. Further analyses identified a positive correlation of circ_SFMBT2 with LATS2. The large tumor suppressor gene (LATS) encodes a ser/thr kinase LATS1 or LATS2 [18]. LATS2 is abnormally expressed in numerous malignancies, including lung, breast, and prostate cancers. LATS2 downregulation could promote cancer cell growth and migration [19]. Particularly, LATS2 was shown to act as a key factor in regulating proliferation, EMT, invasion, and metastatic ability of NSCLC cells [20]. In this study, circ_SFMBT2 overexpression inhibited the expression of LATS2 in the NSCLC cell lines. While cachexia was significantly reduced in cells with an increased expression of circ_SFMBT2, silencing of LATS2 restored the cachexia. In most cases, circ_SFMBT2 was shown to be oncogenic in cancers [21]. The present study demonstrates that circ_SFMBT2 inhibits cancer, showing functional diversity [22].

The article "N6-Methyladenosine Reader YTHDF2 Enhances Non-Small-Cell Lung Cancer Cell Proliferation and Metastasis through Mediating circ_SFMBT2 Degradation" was published in 2022. Journal: Contrast Media Mol Imaging.

LATS2 is considered a vital Hippo/YAP pathway component [23]. The Hippo/YAP pathway is critically involved in organ size control. Multiple studies have found that YAP is upregulated and nuclear-localized in various cancers, while it is capable of promoting stem cell differentiation and renewal during tumor transformation [24]. In particular, while YAP is expressed in NSCLC tissues, YAP overexpression is linked to cancer development and poor prognosis [25]. In addition, YAP could facilitate tumor invasion and metastasis, and drug resistance in NSCLC [26]. In this study, we observed that circ_SFMBT2 overexpression led to a marked upregulation of LATS2 and LATS1, and a significant downregulation of YAP in the cells, while knocking down LATS2 reversed the altered expression of LATS2, LATS1, and YAP in the circ_SFMBT2-overexpressing cells. These observations led us to conclude that circ_SFMBT2 could regulate the malignant behaviors of NSCLC cells presumably by affecting LATS2 expression.

m6A is the most prevalent and reversible post-transcriptional modification in mRNA and circRNA [27]. It has recently been shown to be involved in the metabolism of circRNAs [28]. An m6A reader YTHDF2 binds to its target RNA molecules, and the m6A level in the target RNA can affect the binding between YTHDF2 and its targets [29]. Herein, we showed that while m6A was enriched in circ_SFMBT2, circ_SFMBT2 was significantly upregulated in YTHDF2-knockdown cells. Moreover, RIP and RNA pull-down experiments revealed that YTHDF2 could recognize and bind to circ_SFMBT2. Collectively, these findings proved that both circ_SFMBT2 and YTHDF2 play a key role in NSCLC development.

## 5. Conclusion

This study demonstrated that circ_SFMBT2 was lowly expressed in NSCLC, while it could potentially serve as a biomarker to predict NSCLC development. At the same time, we presented data that YTHDF2 induced the degradation of m6A-modified circ_SFMBT2 and enhanced NSCLC cell proliferation and metastasis by activating the Hippo/YAP pathway. These findings could facilitate our understanding of the effect of m6A modification on circRNA function and mechanisms of NSCLC.

## Figures and Tables

**Figure 1:** circ_SFMBT2 was lowly expressed in NSCLC cells and tissues A and B. Detection of the circ_SFMBT2 level in the paired tumor and normal tissue samples (a) or various NSCLC cell lines as well as HBE cells (b) via qRT-PCR analysis. ^*∗∗*^*p* < 0.01 versus the normal group; ^*∗∗*^*p* < 0.05 versus the HBE group. Nuclear or cytoplasmic expression of circ_SFMBT2 in A549 (c) or H1299 cells (d) was analyzed with qRT-PCR. ^*∗*^*p* < 0.05 versus the nucleus group; ^*∗∗*^*p* < 0.05 versus the nucleus group. (e) Subcellular localization of circ_SFMBT2 was observed by immunofluorescence (scale = 20 *μ*m).

The article "N6-Methyladenosine Reader YTHDF2 Enhances Non-Small-Cell Lung Cancer Cell Proliferation and Metastasis through Mediating circ_SFMBT2 Degradation" was published in 2022. Journal: Contrast Media Mol Imaging.

**Figure 2:** Regulatory effects of circ_SFMBT2 and LATS2 on the NSCLC cell malignancies A and B. Analysis of the expression level of LATS2 in paired tumor and noncancerous tissues (a) or various NSCLC cells as well as HBE cells (b) via qRT-PCR. ^*∗∗*^*p* < 0.01 versus the normal group; ^*∗∗*^*p* < 0.05 versus the HBE group. Determination of circ_SFMBT2 (c) or the LATS2 (d) expression level in the cir_cSFMBT2-overexpressing cells via qRT-PCR. ^*∗∗*^*p* < 0.01 versus the vector group. (e) Pearson's correlation analysis identified a correlation between circ_SFMBT2 and LATS2 expression in the tissues. (f–i) The cell proliferative activity (f), colony-forming ability (g), and migratory ability (h, i) measured using CCK-8 assay, colony formation assay, and transwell assay, respectively. (j) Western blot analysis of MMP-9, E-cadherin, and vimentin expression in the cells. ^*∗∗*^*p* < 0.01 versus the vector group, and ^##^*p* < 0.01 versus the circ_SFMBT2 group.

**Figure 3:** Effects of circ_SFMBT2 in NSCLC cells on the Hippo/YAP pathway. ^*∗∗*^*p* < 0.01 vs the vector group, and ^##^*p* < 0.01 vs the circ_SFMBT2 group.

**Figure 4:** YTHDF2 facilitates the degradation of m6A-modified circ_SFMBT2. (a) The m6A sites in circ_SFMBT2 were predicted using the m6A modification site predictor. (b) The m6A methylation in circ_SFMBT2 was verified by MeRIP. ^*∗*^*p* < 0.01 versus the IgG group. (c) Verification of YTHDF2 knockdown in the cells. (d) Expression analysis of circ_SFMBT2 in YTHDF2 knockdown cells. (e) The binding of circ_SFMBT2 to YTHDF2 was assayed using RNA pull-down experiments. (f) Measurement of circ_SFMBT2 stability in YTHDF2 knockdown cells with qRT-PCR. ^*∗*^*p* < 0.01 versus the siNC group.

**Figure 5:** Effects of circ_SFMBT2 and YTHDF2 on NSCLC progression (a–d). The cell proliferation (a), viability (b), and migratory ability (c, d) were determined using CCK-8 assay, colony-forming assay, and transwell assay, respectively. Western blot analysis of the expression levels of MMP-9, E-cadherin, and vimentin (e) or Hippo/YAP pathway components (f) in the cells. ^*∗∗*^*p* < 0.01 versus the siNC group, and ^##^*p* < 0.01 versus the si-YTHDF2 group.

**Table 1:** The primer sequences.

Targets	DNA sequences (5′ to 3′)
circ_SFMBT2	F: CTGCCAAATTTCCTCTTCCAA
	R: CAACTGTAATGAGGTCTATAGGGCC
LATS2	F: GTTCTTCATGGAGCAGCACGTG
	R: CTGGTAGAGGATCTTCCGCATC
GAPDH	F: GTCTCCTCTGACTTCAACAGCG
	R: ACCACCCTGTTGCTGTAGCCAA

## Data Availability

The data used to support the findings of this study are available from the corresponding author upon request.
